This article has been retracted.

# Establishment and Application of Pressure Injury Assessment Module in Operating Room Based on Information Management System

**DOI:** 10.1155/2022/1463826

**Published:** 2022-01-10

**Authors:** Fangfang Zhou, Zheng Wu, Ying Yu, Lili Xu

**Affiliations:** Operating Theatre, The First Affiliated Hospital of Wenzhou Medical University, Wenzhou 325000, Zhejiang, China

## Abstract

A pressure injury is a common and painful health condition, particularly among people who are elderly or surgical patients. In order to explore how to use the information management system to optimize the pressure injury management process of surgical patients, this work establishes an integrated pressure injury management information platform for surgical patients, which can effectively control the key links in the process and realize the multistep full-process monitoring of surgical patients from admission to discharge. A total of 578 patients before the operation of the information platform were selected as the control group (CG), and after the operation of the information platform, 662 cases became the observation group (OG). Various evaluation metrics are employed to evaluate pressure injury in terms of single-pass rate, high-risk pressure injury, transfer skin condition description matching rate, hospital pressure injury incidence, and incidence of pressure injury in surgical patients at various stages. The results showed that the qualified rate of the pressure injury assessment in the OG was 99.2%, the accuracy rate of high-risk pressure injury screening and reporting was 100.0%, and the matching rate of the transfer skin description was 100.0%, which was higher than that of the CG. The integrated pressure injury management information platform for surgical patients based on the information management system realizes the full, continuous, accurate, and dynamic evaluation and monitoring of patients' skin. Furthermore, it can effectively improve the quality of pressure injury care and facilitate care management.

## 1. Introduction

The development of a pressure injury occurs too frequently in the healthcare setting and adversely affects not only the patient, but also family members, hospital staff, and hospital systems. Direct causes of pressure injuries include shear, friction, amount of pressure, loss of sensation, immobility, and combined pathology [1]. Indirect causes include mobility problems, comorbidities, incontinence, poor nutrition, old age, and psychological health conditions [2]. Many other causes of hospital-acquired pressure injury exist; however, the main cause differs from facility to facility. Patients who are at high risk for pressure injuries are those who are old, immobile, and lacking in proper hydration and nutrition; have neurosensory disorders; use devices that increase skin pressure; and have multiple comorbidities [3].

A pressure injury is caused by severe pressure, continuous pressure, or pressure combined with shear force as shown in Figure 1, which occurs in the skin or the localized damage of the underlying soft tissue under the skin. It mostly occurs in the bone carina or skin [3]. The contact area of medical equipment and other equipment is manifested as the local tissue damage, but the epidermis is open ulcers and may be accompanied by pain. A surgical pressure injury is the local tissue injury caused by the pressure or the combination of pressure and friction or shear force. It is associated with the surgical position and often develops within 72 hours after surgery [4]. Moreover, due to prolonged anesthesia and patients' preoperative physical conditions, surgical patients become a high-risk group of pressure injuries in the hospital. The occurrence of pressure injury not only complicates the treatment of patients but also prolongs the hospital stay and increases the workload of nursing care and medical resources. In the United Kingdom, a huge amount of money is spent on the treatment of pressure injuries each year [5]. In the United States, the annual cost of treating pressure injuries ranges from $9.1 billion to $11 billion, and the personal care of each patient with pressure injury costs $20900–$151700 [6]. The mortality rate in patients with a pressure injury is also significantly higher than in patients without a pressure injury, a 9.1% rate versus a 1.8% rate. In addition to the increased mortality risk, the average hospital charge for a patient with a pressure injury is $36,500, compared to $17,200 for a patient without [7].

The prevention of pressure injuries in surgical patients requires effective nursing measures at all stages of the perioperative period. Therefore, the care of pressure injuries in surgical patients is chain-type, interlocking, and continuous and requires the cooperation of multiple departments. The chained process management refers to the activities that take each link as the management object and maintain the effective continuity of each link as the management purpose [8]. To make all the links in the nursing chain of stress-induced injury closely connected and smooth, based on the characteristics of the integrity of the information transmission of the information system, the convenience of operation, the accuracy of screening, and the real-time monitoring of this project, this work has been established. An integrated pressure injury information platform for surgical patients based on the chain process of the data management system is devised. The system combines different stages of surgical patients to form a preoperation–in-operation–postoperation circulation chain, to stress on surgical and inpatients during hospitalization, standardize the business process of nursing care of sexual injuries, and form a business chain of evaluation–high-risk intervention–handover–nursing, to improve the effectiveness of pressure injury management system.

The rest of the paper is ordered as follows: Section 2 provides a detailed description of the existing pressure injury assessment methods, and section 3 illustrates the proposed research process. In section 4, the different evaluation metrics and the results are presented, and section 5 is about the conclusion.

## 2. Related Work

Pressure injury refers to the localized damage that occurs in the skin and/or underlying soft tissues due to intense and persistent pressure or pressure combined with shear force. It usually occurs in bone carina or skin due to medical equipment or other equipment contacts, showing local tissue damage accompanied by pain [9]. Intraoperative acquired pressure ulcers refer to skin pressure injuries that occur during surgery. There is acute pressure injury that can occur within a few hours or 6 days after surgery, being more common within 3 days after surgery [10]. Surgical patients have become a high-risk group of pressure ulcers in the hospital due to various reasons such as continuous local tissue pressure that cannot be relieved by changing their position, use of surgical auxiliary treatment equipment, long-term anesthesia, and preoperative fasting [11]. The occurrence of intraoperative acquired pressure ulcers not only increases treatment expenses but also requires extensive nursing care [12].

Slowikowski and Funk [13] showed that the incidence of hospital-acquired pressure ulcers within 7 days after surgery can be as high as 14.3%–23.9%. Webster et al. [14] found that 1.3% of surgical patients had a pressure ulcer risk, and more than 1.3% of surgical patients could develop surgery-related pressure ulcers. The study of Scsrlatti et al. [15] showed that the incidence of pressure ulcers in surgical patients reached 20.6% due to the factors of surgical position and operation. A retrospective cohort study [16] found that the incidence of pressure ulcers in surgical patients was 12%. Another systematic literature review in [17] reported that the incidence of pressure ulcers associated with surgery ranged from 0.3% to 57.4%. According to the survey results of Hayes et al. [18], the incidence of pressure ulcers in patients 5 days after surgery can reach 58%.

It has been argued consistently that pressure ulcer risk assessment scales need to be developed based on multivariable analyses to identify factors that are independently associated with pressure ulcer development. Several tools have been developed for the formal assessment of risk for pressure ulcers. To evaluate the pressure ulcer, the Braden Pressure Ulcer Risk Scale was developed by Braden and Bergstrom in the United States in 1987 [19]. It includes six risk factor evaluation indicators: perception, humidity, mobility, nutritional status, friction, and shear force. The scale has a total score of 23 points, of which 15 to 18 are classified as low risk, 13 to 14 are classified as medium risk, 10 to 12 are categorized as high risk, and ≤9 are classified as extremely high risk. This scale is currently one of the most widely used pressure ulcer risk assessment scales, with a sensitivity of 80%–100% and a specificity of 64%–77%. It is suitable for medical and surgical patients and the elderly [20]. He et al. [21] found that the Braden scale has low reliability in predicting pressure ulcers in surgical patients, and it lacks the evaluation of characteristics of surgical patients (such as surgical position, operation time, type of operation, and anesthetic factors). The authors believe that when the Braden scale is used for assessment, it is necessary to combine factors such as the patient's surgical position, time, type, and anesthesia method to accurately evaluate the risk of pressure ulcers in the patient. The Waterlow Pressure Ulcer Risk Scale was developed by Waterlow in 1984 [22]. The scale covers a wider range of pressure ulcer risk factors, including gender, age, body mass index (BMI), and skin type, and also includes operation time, medication, and spinal cord injury. The total score ranges from 4 to 40 points. The higher the score, the higher the risk of pressure ulcers, which can be used for all hospitalized patients. The sensitivity of the scale is 85%–100%, but the specificity is not ideal, 14%–32.9%, and the reliability and internal consistency are low [22]. Although the scale includes the two factors of operation time and major operation, the content of the score appears to be general, and the prediction of pressure ulcers in surgical patients is not accurate enough. The Norton Scale, developed in the United Kingdom, consists of five items: mobility, incontinence, activity, physical condition, and mental condition [23]. Of the several risk factors included in at least one of these three tools, only some factors overlap, specifically mobility, activity, nutrition, incontinence, and cognition. In addition, each scale allocates unique weights to factors, adding to the heterogeneity of the scales. Although several guidelines ratify the use of uniform formal risk assessment tools, the evidence supporting their usage is not clear. A recent update of a Cochrane Collaboration analysis reported only one randomized clinical trial that assessed the impact of a risk assessment tool on the incidence of pressure ulcers [24], and that trial found no effect of the Braden scale on ulcer incidence. A systematic review published in 2006 identified three studies from the 1990s that measured the effect of the Norton Scale on ulcer incidence and also found no effect [25]. This same review described sensitivities ranging from 46.8 to 82.4 and specificities ranging from 27.4 to 67.5 for the Braden, Norton, and Waterlow scales. Generally, usual care will involve the nonformalized use of a risk assessment instrument and will likely vary based on practice patterns and standards. This study takes the pressure injury chain process of surgical patients as the research project, runs it in the pilot operating room, and conducts effect evaluation to ensure the scientific and universal information platform, to gradually extend it to hospitals.

## 3. Material and Methods

### 3.1. General Information

A third-level A hospital in Shanghai, China, and its intensive care unit (ICU) were selected for trial operation of the system in liver surgery. Likewise, cardiothoracic surgery ICU, neurosurgery ICU, operating room, and resuscitation room were also selected to collect data and evaluate the effect. All patients with hospitalization time greater than 24 h were included in this study, and patients undergoing day surgery were excluded.

### 3.2. System Design and Implementation

The system consists of adopting evidence-based nursing methods, raising nursing problems, searching literature, searching scientific basis, evaluating nursing evidence, combined with clinical nursing, and so on, formulating a data management system-based stress injury chain process.  Figure 2 depicts the architecture of the proposed system.

#### 3.2.1. Design of Hospital Circulation Chain

The pressure injury management of surgical patients is a care transfer chain, including the entire process “before surgery–during surgery–after surgery.” The transfer of patients involves multiple departments such as the ward, operating room, recovery room, and ICU. Therefore, the management of pressure injury in surgical patients is also a multisectoral process. In the process of multidepartmental information transmission, there may be inconsistencies in records such as evaluation, risk screening, and skin integrity, or due to lack of effective communication between departments, when considering the risk of stress injury, only current factors are considered, and some continuations are ignored such as sexual factors. Due to the different international scales for postadmission-preoperative-postoperative evaluation of patients, most of the current domestic information systems for stress injury only focus on one stage of the patient's hospitalization process or separate the evaluation records of the same patient according to different stages of hospitalization. For nurses in the operating room to understand the evaluation of the preoperative ward, they need to click on different links to inquire. The final form is also isolated. From the preoperative and intraoperative point of view, it is impossible for us to intuitively understand the admission of patients. We use the characteristics of complete information transmission in the information system to conduct a chain combination of the evaluation and records (including risks, incision conditions, compressed parts, and nursing measures) of the departments involved in the preoperative-intraoperative-postoperative flow chain of surgical patients. The information can be displayed intuitively and accurately on the same interface, so as to realize multiteam cooperation in stress injury management.

#### 3.2.2. Design of Nursing Business Chain for Pressure Injury

The entire business chain of pressure injury care for surgical patients includes evaluation, high-risk intervention, handover, and nursing care. High-risk patients are screened out by evaluating the patients' pressure injury risk factors, and effective precontrol measures are taken to identify the patients' high-risk factors and follow-up. The management opinions are passed to the next link of the perioperative period, and the follow-up departments conduct predictive management and take personalized nursing measures. These processes are explained as follows.

- Evaluation: according to the different predisposing factors of pressure injury after admission and perioperative period of patients in the operating department, an appropriate scale is selected in a targeted manner that also includes the device-induced injury into the scope of the evaluation. By evaluating the predisposing factors of pressure injury and skin condition, patients with a high risk of pressure injury are screened out, as shown in Figure 3. The continuous risk assessment in the process of patient circulation can be regarded as continuous clinical observation and judgment of the patient's pressure injury risk, to take preventive measures that meet specific risk factors. In the information platform, the nurse can click on the current evaluation department, and the system can identify high-risk patients based on the definition of the high-risk score on the evaluation scale. For patients with preexisting pressure injuries, the default is high-risk patients. To monitor the timeliness of the evaluation, the background system compares the actual evaluation time and screens outpatients whose evaluation is greater than 2 hours, to enable the management staff to monitor and assess the timeliness of the assessment in each ward.
- High-risk intervention: based on the evaluation and screening results, evidence-based preventive skin management strategies are adopted for high-risk patients before, during, and after surgery. High-risk patients are included in the third-level monitoring system of the head nurse nursing department after reporting according to the system requirements. Using the information system, the reported status is divided into nine states (three high-risk prediction states and six occurrence states) according to the patient's high-risk situation. The structure model established in the background analyzes and calculates the reporting status and automatically jumps to the reporting status. The management interface realizes a three-level monitoring function, forming a summary of the jurisdiction area according to the identity of the user who login in and sorted and filtered according to requirements, which is convenient for management personnel at all levels to check bottom-up layer-by-layer reporting function and top-down monitoring and guidance function to realize interaction.
- Handover: patient stress injury management is a continuous process. During cross-departmental handover, the preoperative patient's skin condition, special circumstances, follow-up management suggestions, and precautions must be completely and correctly transmitted to establish a good interdepartmental relationship. This communication helps follow-up departments to accurately grasp the status of patients and take effective measures. In the handover link, the preoperative department and the operating room need to complete the preoperative high-risk factors and early warning of the patient. The postoperative operating room nurse will promptly hand over the patient's high-risk factors during the operation to the resuscitation room and subsequent departments. This can help nurses and managers analyze possible causes of injury and implement process improvements. The content that needs to be handed over is embedded in the nursing form through the information platform, and it can be saved after it is filled in completely. After the system completes the transfer of departments, the handover information is automatically displayed. After the receiving department completes the handover, it is confirmed on the information platform, and the handover process and content are standardized.
- Nursing: the nursing of pressure injuries in surgical patients is an ongoing process. The nurses in the follow-up department should correctly identify the pressure injury and ensure the continuous decompression of the compressed area; at the same time, within 24 hours after surgery, the surgical nurse should enter the ward and ICU for a return visit to assess the skin condition of the compressed area during the operation. In the event of a stress injury, the operating room should be notified in time, the adverse event should be reported, the cause analysis should be performed, the cause of the injury should be analyzed, and process improvement should be implemented. In the information platform, use of decompression pads, selection of reasonable supports, postoperative decompression methods, incision treatment, and other nursing measures are standardized and set for nurses to check. In the background monitoring, patients with postoperative pressure injury are screened out, and the pressure site during the operation is compared with the site where the pressure ulcer occurs, as one of the bases for confirming the pressure injury related to the operation; the postoperative pressure injury healing time is counted as a reference for the effectiveness of nursing measures. The occurrence of stress injuries is automatically included in the adverse event reporting system.

### 3.3. Statistical Analysis

SPSS 21.0 statistical software was used for data analysis. Measurement data are expressed in the form of mean ± standard deviation, comparison between groups is accomplished with the help of *t*-test, count data is expressed by frequency and percentage, and comparison between groups is by expressed by *χ*^2^ test and Fisher's exact test. The rank data is represented by rank-sum test. The difference was considered statistically significant when *P* < 0.05 and insignificant otherwise.

## 4. Experiment and Discussion

### 4.1. Data Information

A third-level A hospital in Shanghai, China, was selected for data collection. For the trial operation of the system, patients with liver surgery, cardiothoracic surgery, neurosurgery and their ICUs, operating room, and resuscitation room were selected to evaluate the effect. The cluster sampling method was used to select 1,240 inpatients in the operating department as the research objects. Among them, 578 patients before the operation of the information platform were selected as the control group, and 662 patients after the operation of the information platform were chosen as the observation group. In the observation group, there were 451 males and 211 females with an average age of 52.1 ± 16.8 years. Among the 662 patients, 339 were surgical patients including 188 males and 151 females, with an average age of 50.6 ± 18.4 years and an average operation time of 3.5 ± 1.9 hours. The control group included 386 males and 192 females, with an average age of 50.2 ± 19.2 years. Among the total patients of the control group, 292 were surgical patients with 175 males and 117 females, with an average age of 52.4 ± 18.4 years and an average operation time of 3.6 ± 2.1 hours. There was no statistically significant difference in the general information of the two groups of patients, and they were comparable.

### 4.2. Evaluation Metrics

The data about the control group was obtained by checking the medical record, and the observation group data was obtained by the information system. The different evaluation metrics for inpatients and surgical patients are discussed as follows.

The general evaluation indices for inpatients are computed as follows:

- The qualified rate of the pressure injury evaluation sheet for inpatients = the number of qualified cases for the pressure injury evaluation sheet/the total number of cases for the examination evaluation sheet × 100%.
- The accuracy of screening and reporting high-risk pressure injury hospitalized patients = the actual number of reported cases of high-risk pressure injury hospitalized patients/the number of high-risk pressure injury hospitalized patients that should be reported × 100%.
- The accuracy of screening and reporting of patients with pressure injury = the actual number of reported cases of patients with pressure injury/the number of cases that should be reported for patients with pressure injury × 100%.
- The incidence of pressure injury in hospital = the number of new cases of pressure injury in the hospital during the cycle/total number of hospitalized patients in the cycle × 100%.

The specific evaluation indices for surgical patients are as follows:

- The matching rate of the description of the skin condition of the surgical patient's transfer = the number of matching cases with the description of the skin condition of the surgical patient's transfer/the total number of patients undergoing inspection × 100%.
- Determining that the description of the skin condition of the transfer is consistent, the skin condition described in the skin assessment sheet record of the two departments at the time of the transfer is deemed to be consistent.
- The incidence of hospital pressure injury in surgical patients = the number of new cases of hospital pressure injury in surgical patients during the cycle/total number of surgical patients in the cycle × 100%.
- The incidence of stage 1 pressure injury in surgical patients = the number of new cases of stage 1 pressure injury in surgical patients during the cycle/total number of surgical patients in the cycle × 100%.
- The incidence of stage 2 pressure injury in surgical patients = the number of new cases of stage 2 pressure injury in surgical patients during the cycle/total number of surgical patients in the cycle × 100%.

### 4.3. Comparison of General Evaluation Indicators for Patients

Figure 4 shows the qualification rate of the pressure injury assessment documents. The qualified rate of the pressure injury assessment documents of the patients before and after the use of the information platform was 92.2% and 99.2%, respectively, and the difference between the two groups was statistically significant (*P* < 0.05). The comparison of the accuracy rate of screening and reporting of high-risk pressure injury for inpatients in the operating department of the two groups is shown in Figure 5. The accuracy rate before the use of the information platform was 97.3% and after the application of the information system was 100.0%, with prominent statistical differences. Likewise, the comparison of the incidence of pressure injury in the two groups of inpatients in the operating department is represented in Figures 6 and 7. The information platform was 3.3% before use and 1.5% after use.

### 4.4. Comparison of Matching Rate of Skin Condition Description for Patients

We compared the matching rate of skin conditions for different patients. The matching rate of the information platform was 91.4% before use and 100% after use, showing that the difference was statistically significant. While comparing the incidence of pressure injury in hospitals between the two groups of surgical patients, we found that the recognition rate of the information platform was 6.5% before use and 3.0% after use. We also compared the incidence of stage 1 pressure injury between the two groups of surgical patients. The incidence of stage 1 pressure injury before the use of the information platform was 5.8% and after the use was 2.7%, which shows that the results are statistically significant (*P* < 0.05).  Table 1 shows the incidence of stage 1 pressure in different groups. In Table 1, CG is the control group. OG is an observation group, and STTSD represents the surgical transfer and transfer of skin description. OS1PISP is the occurrence of stage 1 pressure injury in surgical patients. OS2PISP is the occurrence of stage 2 and above pressure injuries in surgical patients.

## 5. Conclusion

With the increased focus on patient safety and quality of care, understanding how to prevent pressure injury has become a primary interest in acute care hospitals. This study is based on the data management system chain process of the surgical patient pressure injury information platform to achieve the full evaluation of patients from admission to discharge, identify high-risk patients, and timely implement intervention measures, in addition to the continuity of nursing measures through the improvement of handover links. A total of 578 patients were selected as CG, and 662 cases became the OG. The results of the two groups were compared in terms of matching rate, hospital pressure injury incidence, and incidence of pressure injury in surgical patients. The results showed that the proposed information management system can effectively improve the quality of evaluation documents, ensure the accuracy of screening and reporting, guarantee the correctness of skin handover, and reduce the incidence of pressure injuries. It is not only suitable for surgical patients but also widely used in the management of stress injuries for all hospitalized patients. It realizes the whole process and provides continuous, accurate, and dynamic evaluation and monitoring of patients' skin, which has certain application value. This work has important clinical significance for reducing the suffering of patients and improving the quality of life of patients.

## Figures and Tables

**Figure 1:** The pressure injury.

**Figure 2:** Chain flow chart of stress injury based on the data management system.

**Figure 3:** Evaluation and screening flow chart.

**Figure 4:** The quality of stress injury assessment document.

**Figure 5:** Screening of patients with a high-risk pressure injury.

**Figure 6:** The screening of patients with a stress injury.

**Figure 7:** The occurrence of pressure injuries in the hospital.

**Table 1:** Comparison of specific evaluation indicators.

Group	Operation number	STTSD		OS1PISP		OS2PISP		OPISP	
		QN	PR	ON	OR	ON	OR	ON	OR
CG	292	268	91.4	18	5.8	2	0.7	20	6.5
OG	339	339	100.0	9	2.7	1	0.3	10	3.0
*χ* ^2^	—	30.2		4.0		4.2		4.6	
*P*	—	0.001		0.044		0.600		0.035	

OPISP is the occurrence of pressure injury in surgical patients. QN is the number of qualified cases. PR shows the pass rate, ON is the number of occurrences, and OR indicates the occurrence rate. It can be seen that the ON and OR for the CG are greater than the OG for STTD, OSIPISP, OS2PISP, and OPISP. Moreover, the results are significant (*P* < 0.05) in all cases.

## Data Availability

The datasets used and analyzed during the current study are available from the corresponding author upon reasonable request.
